# Exploring the Temporal Correlation of Sarcopenia with Bone Mineral Density and the Effects of Osteoblast-Derived Exosomes on Myoblasts through an Oxidative Stress–Related Gene

**DOI:** 10.1155/2022/9774570

**Published:** 2022-09-15

**Authors:** Jingsong Chen, Jie Shen, Xili Yang, Huiting Tan, Ronghua Yang, Cuiying Mo, Ying Wang, Xiaojun Luan, Wenhua Huang, Guoqiang Chen, Xuejuan Xu

**Affiliations:** ^1^Department of Endocrinology, The First People's Hospital of Foshan, Foshan, Guangdong 528000, China; ^2^Department of Endocrinology, Shunde Hospital of Southern Medical University (The First People's Hospital of Shunde), Foshan, Guangdong 528399, China; ^3^Department of Cardiology, The First People's Hospital of Foshan, Guangdong 528000, China; ^4^Department of Burn and Plastic Surgery, Guangzhou First People's Hospital, South China University of Technology, Guangzhou, Guangdong, China; ^5^Department of Nuclear Medicine, The First People's Hospital of Foshan, Foshan, Guangdong 528000, China; ^6^Guangdong Engineering Research Center for Translation of Medical 3D Printing Application, Guangdong Provincial Key Laboratory of Medical Biomechanics, National Key Discipline of Human Anatomy, School of Basic Medical Sciences, Southern Medical University, Guangzhou, Guangdong 510515, China; ^7^Guangdong Medical Innovation Platform for Translation of 3D Printing Application, The Third Affiliated Hospital of Southern Medical University, Guangzhou, Guangdong 510000, China; ^8^Department of Rheumatology, The First People's Hospital of Foshan, Foshan, Guangdong 528000, China

## Abstract

Sarcopenia is an age-related accelerated loss of muscle strength and mass. Bone and muscle are closely related as they are physically adjacent, and bone can influence muscle. However, the temporal association between bone mineral density (BMD) and muscle mass in different regions of the body after adjustment for potential indicators and the mechanisms by which bone influences muscle in sarcopenia remain unclear. Therefore, this study aimed to explore the temporal association between muscle mass and BMD in different regions of the body and mechanisms by which bone regulates muscle in sarcopenia. Here, cross-lagged models were utilized to analyze the temporal association between BMD and muscle mass. We found that low-density lipoprotein (LDL-C) positively predicted appendicular lean mass. Mean whole-body BMD (WBTOT BMD), lumbar spine BMD (LS BMD), and pelvic BMD (PELV BMD) temporally and positively predicted appendicular lean mass, and appendicular lean mass temporally and positively predicted WBTOT BMD, LS BMD, and PELV BMD. Moreover, this study revealed that primary mice femur osteoblasts, but not primary mice skull osteoblasts, induced differentiation of C2C12 myoblasts through exosomes. Furthermore, the level of long noncoding RNA (lncRNA) taurine upregulated 1 (TUG1) was decreased, and the level of lncRNA differentiation antagonizing nonprotein coding RNA (DANCR) was increased in skull osteoblast–derived exosomes, the opposite of femur osteoblast–secreted exosomes. In addition, lncRNA TUG1 enhanced and lncRNA DANCR suppressed the differentiation of myoblasts through regulating the transcription of oxidative stress–related *myogenin* (*Myog*) gene by modifying the binding of myogenic factor 5 (Myf5) to the *Myog* gene promoter via affecting the nuclear translocation of Myf5. The results of the present study may provide novel diagnostic biomarkers and therapeutic targets for sarcopenia.

## 1. Introduction

Sarcopenia is an age-related accelerated loss of muscle strength and mass in older individuals. It increases the risk of falls, fractures, functional decline, and frailty and leads to considerable healthcare costs, poor quality of life, and mortality [1, 2]. Sarcopenia is common among older adults, and the incidence of sarcopenia is increasing rapidly [3]. Although antioxidant and pharmacological agents, including myostatin and activin, have been utilized to treat skeletal muscle atrophy and dysfunction, some studies have reported the off-target effects of these drugs [4, 5]. Thus, research related to age-related (primary) sarcopenia and disease-related (secondary) sarcopenia has focused on improving diagnosis and therapy, with special interest in exploring diagnostic biomarkers and targets for drugs of resistance exercise [3, 6].

In the musculoskeletal system, bone and muscle are closely related as they are physically adjacent. Among age-related diseases, sarcopenia is strongly associated with osteoporosis [7, 8]—a common skeletal disorder caused by a decline in muscle mass [9]. Therefore, bone can exert influence on muscle. Recent studies have focused on the relationship between muscle mass and BMD. For instance, a recent study has revealed that reduced BMD correlates with decreased muscle mass and strength in Chinese subjects with sarcopenia [10]. Our recent study indicated that skull BMD negatively correlates with appendicular skeletal muscle (ASM) mass, whereas BMDs throughout the rest of the body are positively associated with ASM mass in male middle-aged and elderly Chinese individuals [11]. However, the temporal association between sarcopenia (muscle mass) and BMD in different regions of the body after adjustment for potential indicators including albumin, F-box protein 2 (FBXO2/FBS), LDL-C, thyroid-stimulating hormone (TSH), and platelet distribution width remains unclear.

To date, the knowledge on mechanisms by which bone influences muscle is still limited. It is considered that bone and muscle communicate with each other in a paracrine and endocrine manner, and there are various collaborative changes between these two tissues induced by numerous biochemical signals or weight-bearing stimulation [12]. For instance, osteoblast-derived osteoglycin (OGN) may play a role in regulating muscle mass [13]. In addition, the level of prostaglandin E2 secreted by bone cells is much higher than that secreted by damaged muscle cells, which is conducive to muscle regeneration and repair [13]. Extracellular vesicles, including microvesicles and exosomes, are vesicles secreted by cells and mediate the communication among different cells and organs [14]. However, the effect of exosomes derived from osteoblasts on myoblasts is largely unknown.

Exosomes could mediate long-distance communication and cooperative regulatory network among different cells and organs as vectors to carry long noncoding RNAs (lncRNAs) in a variety of diseases [15–17]. Previous studies have shown that lncRNA TUG1 promotes the osteogenic differentiation of osteoblasts through suppressing the Wnt/*β*-catenin pathway [18]. In contrast, lncRNA DANCR inhibits osteogenic differentiation by activating the Wnt/*β*-catenin pathway [19]. However, the roles of lncRNA TUG1 and DANCR in myoblasts or muscle have not been reported. Surprisingly, the prediction of RNA–protein binding by RPISEQ (http://pridb.gdcb.iastate.edu/RPISeq/index.html) showed that both lncRNA TUG1 and DANCR had high binding probability with Myf5 (Supplementary Figure S1), suggesting that lncRNA TUG1 and DANCR in osteoblasts-derived exosomes might play critical roles in myoblasts or muscle.

Our latest study has revealed that the relationships between muscle mass and different bone tissues are different [9], suggesting that exosomal lncRNAs derived from different osteoblasts might exert different regulatory effects on muscle mass. Therefore, this study aimed to explore the temporal association between sarcopenia (muscle mass) and BMD in different regions of the body and the effects of exosomal lncRNA TUG1 and DANCR derived from different osteoblasts on myoblasts.

## 2. Methods and Materials

### 2.1. Participants

A total of 3179 male individuals (30–100 years old) with complete body composition and data whole-body BMD detected by the Health Care Department of Foshan First People's Hospital from 2014 to 2016 were recruited for this study. Based on medical history and examination results, we excluded individuals with complete loss of walking ability; alcoholism (more than 210 g per week); other chronic liver diseases; viral or autoimmune hepatitis; severe cardiac or renal insufficiency or severe dementia (MMSE <18 points); use of steroids or immunosuppressants; autoimmune diseases; use of drugs or items that may affect body weight and body composition; pathological obesity; uncontrolled diabetes; or hypothyroidism and other endocrine/metabolic diseases diagnosed in the past five years. The current study was approved by the Ethics Committee of Foshan First People's Hospital, and written informed consent was obtained from each participant.

### 2.2. Measurement of BMD

BMD of the whole body (mean value), head, femoral neck, thoracic spine, left upper arm, right upper arm, lumbar spine, left leg, right leg, left rib, right rib, pelvis, and hip was measured using dual-energy X-ray absorptiometry (DXA, HOLOGIC, Marlborough, MA, USA). The absorptiometry was calibrated daily utilizing the model provided by the manufacturer to maintain the stability of measurement. The coefficient of variation (percentage) of repeated measurements met the accurate criteria of femoral neck (2.5%), lumbar spine (<1.9%), and total femur (<1.8%). Moreover, the values of total and regional BMD (g/cm^2^) were identified by DXA using standard procedures. Next, BMD values were classified by WHO criteria based on *T* values of femoral neck and/or lumbar spine and/or hip as follows: normal population (*T* value> −1.0 SD), bone mass reduction (−1.0 SD ≤ *T* value ≤ −2.5 SD), and osteoporosis (*T* value ≤ −2.5 SD).

### 2.3. Detection of Muscle Mass

Muscle mass was detected using DXA (HOLOGIC), and sarcopenia was diagnosed according to two definitions: (1) appendicular skeletal muscle index (ASMI): the mass of appendicular skeletal muscle divided by the square of height (kg/m^2^), with the threshold of 7.0 kg/m^2^ in males; and (2) skeletal muscle index (SMI): the percentage of skeletal muscle mass of limbs in body weight, with the threshold of 29.9% in males. In this study, male subjects with ASMI <0.7 or SMI<29.9% were defined as “early sarcopenia” and recruited.

### 2.4. Measurement of Blood Biochemical Metabolic Indexes

After more than 8 hours of fasting, forearm venous blood was taken from the subjects between 8 a.m. and 10 a.m., and the subjects sat. Blood processing and collection were performed under strictly standardized conditions. Subsequently, serum albumin was analyzed by turbidimetry, and the coefficient of variation was 2%. FBS, LDL-C, TSH, and platelet distribution width were evaluated using an Olympus AU5400 Automatic Biochemical Analyzer (Tokyo, Japan).

### 2.5. Analytic Plan

Continuous variables were presented using means ± standard deviation (SD), and categorical variables were described as a percentage (%). We used a *t* test or ANOVA to estimate the differences in BMDs depending on demographic characteristics and other variables. Pearson correlation analyses were used to analyze the intercorrelations among muscle mass and BMDs across different investigations. A series of structural equation models with autoregressive cross-lagged design (ACLD) were used to estimate the temporal associations among muscle mass and BMDs after adjustment for potential confounders, including albumin, FBS, LDLC, TSH, and platelet distribution width. ACLD has been demonstrated to be a useful method for examining potential associations between two variables over time (https://www.tandfonline.com/loi/wean20). Here, we hypothesized the bidirectional relation of BMDs and muscles mass, that is, that higher BMDs may lead to more muscle mass and that more muscle mass may reversely result in higher BMDs. To test our hypotheses, three models were developed. Model 1 was applied to examine the temporal effects of BMDs or muscle mass at time *T*-1 on BMDs or muscle mass at time *T*; model 2 was applied to test the effects of BMDs at time *T*-1 on muscle mass at time *t* and the effects of muscle mass at time *T*-1 on BMDs at time *T*; and model 3 was a combination of model 1 and model 2. We reported standardized regression coefficients in all structural equation models. Associations were analyzed by Package for the Social Sciences software (v 20.0) (SPSS Inc., Chicago, Illinois, USA) and Analysis of Moment Structures (AMOS) (v 20.0). All of the tests that were conducted were two-sided. The overall model fit was evaluated using the root-mean-square error of approximation (RMSEA, <0.08) and the comparative fit index (CFI, >0.90).

### 2.6. Cell Culture

Primary mice osteoblasts of skull, primary mice osteoblasts of femur, and C2C12 cells were purchased from LANDM Biotech (Guangzhou, Guangdong, China). All cells were cultured with DMEM high glucose medium (Hyclone, Logan, UT, USA) containing 100 units/mL penicillin (Hyclone) and 10% fetal bovine serum (Hyclone) in a 37°C atmosphere filled with 5% CO_2_ [20].

### 2.7. Cell Treatment

The differentiation of C2C12 cells was induced by DMEM high glucose medium (Hyclone) with 2% horse serum (Bioind, Kibbutz Beit Haemek, Israel) (differential medium). To identify the effect of osteoblasts on myoblasts, culture media of primary mice osteoblasts of skull and primary mice osteoblasts of femur were collected to culture C2C12 cells combined with C2C12 cell culture medium (0%, 50%, or 100%). Moreover, C2C12 cells were incubated with exosomes isolated from the culture media to identify the effects of exosomes derived from osteoblasts on C2C12 cells. In addition, transfection of vectors was performed using Lipofectamine 2000 (Invitrogen, Carlsbad, CA, USA).

### 2.8. Cell Counting Kit-8 (CCK8) Assay

First, C2C12 cells were seeded in 96-well plates at the concentration of 1 × 10^4^/mL. After the indicated treatments, 10 *μ*L CCK8 solution (Beyotime, Shanghai, China) at a 1/10 dilution was added to incubate C2C12 cells at 37°C for 1.5 h [21]. Then, absorbance at 450 nm was assayed using a Multiscan MK3 (Thermo Fisher Scientific, Waltham, MA, USA). The means of the optical density (OD) were used to calculate the cell proliferation rate according to the following formula: Cell proliferation rate (%) = (OD treatment group/OD control group) × 100%.

### 2.9. Apoptosis Assay

A total of 1 × 10^6^ C2C12 cells of each group were collected and washed twice using the incubation buffer containing 10 mmol/L HEPES/NaOH (pH 7.4), 140 mmol/L NaCl, and 5 mmol/L CaCl_2_ [22]. Next, C2C12 cells were resuspended in 150 *μ*L of phosphate-buffered solution (PBS) including 1.5 *μ*g/mL Annexin V (KeyGen, Nanjing, Jiangsu, China) and propidium iodide (PI) (Thermo Fisher Scientific). Then, the cells were incubated with Annexin V and PI in dark at room temperature (RT) for 15 min. After washing with PBS, C2C12 cells were resuspended again in 400 *μ*L incubation buffer and analyzed using flow cytometry (BD FACSCalibur, BD Biosciences, San Jose, CA, USA).

### 2.10. Detection of Oxidative Stress

To detect oxidative stress in C2CC12 cells, the levels of malondialdehyde (MDA), L-glutathione (GSH), and superoxide dismutase (SOD) were identified. MDA level was identified using Lipid Peroxidation MDA Assay Kit (#S0131S) purchased from Beyotime. GSH level was tested by Micro Reduced Glutathione (GSH) Assay Kit (#BC1175) obtained from Solarbio (Beijing, China). SOD level was measured utilizing Superoxide Dismutase Activity Assay Kit (#BC0170) from Solarbio. Detections were performed in accordance with the manufacturers' instructions.

### 2.11. Western Blot (WB)

Total proteins were first extracted from C2CC12 cells or exosomes. Then, the same amount of protein (40 *μ*g) was loaded into SDS-polyacrylamide gel and separated using electrophoresis. Next, the proteins were transferred onto PVDF membranes (Millipore, Bedford, MA, USA) and blocked with 5% nonfat milk for 1 h at RT. Subsequently, the membranes were incubated with primary antibodies at 4°C overnight with gentle shaking [11, 23]. After incubation with primary antibodies, the membranes were washed with Tris-buffered saline containing 0.1% Tween20 (TBST) and then incubated with corresponding secondary antibodies (1 : 5000, Southern Biotech, Birmingham, AL, USA) at RT for 1 h [9, 23]. Finally, signals of the targeted proteins were detected using Immobilon Western Chemilum HRP Substrate (Millipore). The primary antibodies used in this study included MYH6 antibody (1 : 500, Abcam, Cambridge, MA, USA), Myog antibody (1 : 200, Abcam), myHC antibody (1 : 500, Abcam), CD63 antibody (bs-1523R, Bioss, Beijing, China), CD81 antibody (bs-6934R, Bioss), and GAPDH antibody (1 : 3000, Kangcheng, Shanghai, China).

### 2.12. Isolation and Analysis of Exosomes

GS™ Exosome Isolation Kit (for cell culture media) (E5001, Geneseed, Guangzhou, Guangdong, China) was used to isolate exosomes in accordance with the manufacturer's instruction. To further confirm that exosomes were isolated, their morphology was detected utilizing transmission electron microscopy (TEM) (HT-7700, Hitachi, Tokyo, Japan), and the size was identified using nanoparticle tracking analysis (N30E, NanoFCM, Nottingham, UK). Moreover, the markers of exosomes, including CD63 and CD81, were detected by WB.

### 2.13. Quantitative Real-Time PCR (qPCR)

Total RNA from C2C12 cells or exosomes was extracted by TRIzol (Invitrogen). Then, RNA was reverse-transcribed to cDNA using PrimeScript II 1st Strand cDNA Synthesis Kit (Takara Biotechnology, Dalian, Liaoning, China). Next, qPCR was performed by CFX96 Touch Real-Time PCR (Bio-Rad, Hercules, CA, USA) utilizing SYBR Premix Ex Taq II (Takara Biotechnology). Subsequently, the amount of target RNA was normalized to that of GAPDH (internal control), and the fold change of target RNA was identified by 2^-△△Ct^ relative to the control group [11, 23]. The sequences of primers used for qPCR were as follows: Myf5 forward: 5′-GCATCTACTGTCCTGATGTA-3′, reverse: 5′-CATCGGGAGAGAGTTCATAA-3′; lncRNA TUG1 forward: 5′-TATTGGTATGGCTGGCCTTTC-3′, reverse: 5′-TGGGTGAGGTGTGGGTTGTT-3′; lncRNA DANCR forward: 5′-CAGTTCTTAGCGCAGGTTGA-3′, reverse: 5′-AGCATTGTCACTGCTCTAGCT-3′; GAPDH forward: 5′-GGCCTCCAAGGAGTAAGAAA-3′, reverse: 5′-GCCCCTCCTGTTATTATGG-3′.

### 2.14. RNA Immunoprecipitation (RIP) Assay

The RIP assay was performed using an EZ-Magna RIP kit (Millipore). Lysates were obtained from 1 × 10^7^ C2C12 cells using complete RIP lysis buffer and then immunoprecipitated with RIP buffer containing conjugated magnetic beads (Abcam) and anti-Myf5 antibody. Next, the precipitated RNAs with Myf5 protein were detected by qPCR. Rabbit IgG was used as the negative control.

### 2.15. Luciferase Reporter Gene System

First, the *Myog* gene promoter was cloned into the luciferase reporter gene plasmid. Then, C2C12 cells were cotransfected with the luciferase reporter gene plasmid and the lncRNA TUG1 expression vector or the lncRNA DANCR expression vector. After transfection for 48 h, C2C12 cells were collected to detect the relative luciferase activity using a dual-luciferase reporter assay system (Promega, Fitchburg, Wisconsin, USA).

### 2.16. Chromatin Immunoprecipitation (ChIP)

A ChIP kit obtained from Thermo Fisher Scientific was utilized to assess ChIP. In brief, C2C12 cells were cross-linked by 1% formaldehyde at RT for 15 min and then stopped by glycine. Then, C2C12 cells were sonicated to shear DNA. Next, 25 mg DNA chromatin sample was diluted by 450 mL dilution buffer with protease inhibitors. Subsequently, chromatin samples were incubated with 1 *μ*g Myf5 antibody (Abcam)/antirabbit IgG antibody (Abcam) and magnetic protein A/G beads at 4°C with gentle rotation overnight. After incubation, the magnetic beads were collected using magnetic separation device (Thermo Fisher Scientific) and cleaned. Subsequently, 100 *μ*L elution buffer containing proteinase K was utilized to elute immunoprecipitated DNAs at 62°C for 2 h. Then, the immunoprecipitated DNAs were purified using the spin columns. Finally, chromatin DNAs were analyzed by qPCR. Primers used for ChIP-qPCR in the present study were as follows: Myog ChIP1 forward: 5′-CTGTTGCCCGTGCCGGAGCG-3′, reverse: 5′-AGAATTTGGCCAGATGCAGTG-3′; Myog ChIP2 forward: 5′-GCCCAAACTTCATGATGTCTC-3′, reverse: 5′-AAGAATTTTCCAGGCAGGCC-3′; Myog ChIP3 forward: 5′-CGTCTCCCCAATACGATGTTATG-3′, reverse: 5′-CTCCCCTCCAAGAAAGGGCCAC-3′; Myog ChIP4 forward: 5′-ATCATGGTTCATTGGCAGCC-3′, reverse: 5′-CAGGCACAGTGACTCATGCC-3′.

## 3. Statistical Analysis

All quantitative data were presented as mean ± SD. Experiments in this study were repeated three times (*n* = 3). Next, statistical differences were analyzed by SPSS 20 software (SPSS Inc., Chicago, IL, USA). Briefly, the unpaired Student's *t*-test was used to compare two groups, while one-way ANOVA was utilized for comparisons among multiple groups. *P* < 0.05 was considered statistically significant.

## 4. Results

### 4.1. Clinicopathological Features of Patients with Sarcopenia

The clinicopathological features of 384 male patients with sarcopenia are described in Table 1. Briefly, their median age was 51.6 years (33–93 years); median weight was 72.7 kg (51.9–102.6 kg); median height was 170.5 cm (145–184 cm); and median body mass index (BMI) was 25.0 (16.8–33.6) at T1 (the first year of this study). These clinicopathological features were consistent at each measurement time, including T1 (the first year of this study), T2 (the second year of this study), and T3 (the third year of this study).

### 4.2. Descriptive Statistics

The mean values for the analyzed variables at each measurement time are presented in Table 2. The average values of appendicular lean mass, mean whole-body BMD (WBTOT BMD), skull BMD (HEAD BMD), lumbar spinal BMD (LS BMD), and pelvic BMD (PELV BMD) were 8.07 (5.93–10.52), 1.12 (0.91–1.42), 2.19 (1.44–3.01), 1.00 (0.65–1.52), and 1.24 (0.91–2.08) at T1, respectively. Moreover, the median values at T1 of albumin-1, FBS, LDL-C, TSH, and platelet distribution width were 43.47 *μ*g/mL (35.9–45.7 *μ*g/mL), 5.29 *μ*g/mL (3.69–13.72 *μ*g/mL), 2.94 *μ*g/mL (0.77–5.2 *μ*g/mL), 1.77 *μ*g/mL (0.01–13.26 *μ*g/mL), and 13.44 (8.88–21.2), respectively. Except for platelet distribution width, other clinicopathological features were consistent from T1 to T3. Appendicular lean mass, WBTOT BMD, HEAD BMD, LS BMD, and PELV BMD were consistent at each measurement time (T1 to T3).

### 4.3. Cross-Lagged Paths between WBTOT BMD and Appendicular Lean Mass

Albumin-1, FBS, LDL-C, TSH, and platelet distribution width were used as covariates. The model including cross-lagged paths between WBTOT BMD and appendicular lean mass did not fit the data well (RMSEA = 0.45; CFI = 0.04). As shown in Figure 1(a), LDL-C at T1 positively predicted T1 appendicular lean mass. WBTOT BMD at T1 positively predicted T2 appendicular lean mass, while WBTOT BMD at T2 positively predicted T3 appendicular lean mass (Figure 1(a)). Furthermore, appendicular lean mass at T1 positively predicted T2 WBTOT BMD, and appendicular lean mass at T2 positively predicted T3 WBTOT BMD (Figure 1(a)).

### 4.4. Cross-Lagged Paths between HEAD BMD and Appendicular Lean Mass

The model including cross-lagged paths between HEAD BMD and appendicular lean mass did not fit the data well (RMSEA = 0.406; CFI = 0.002). Platelet distribution width at T1 negatively predicted T1 HEAD BMD (Figure 1(b)). However, HEAD BMD did not predict appendicular lean mass (Figure 1(b)).

### 4.5. Cross-Lagged Paths between LS BMD and Appendicular Lean Mass

The model including cross-lagged paths between LS BMD and appendicular lean mass did not show a good fit (RMSEA = 0.424; CFI = 0.03). As shown in Figure 2(a), LDL-C at T1 positively predicted T1 appendicular lean mass. LS BMD at T1 positively predicted T2 appendicular lean mass, while LS BMD at T2 positively predicted T3 appendicular lean mass (Figure 2(a)). Furthermore, appendicular lean mass at T1 positively predicted T2 LS BMD, and appendicular lean mass at T2 positively predicted T3 LS BMD (Figure 2(a)).

### 4.6. Cross-Lagged Paths between PELV BMD and Appendicular Lean Mass

The model including cross-lagged paths between PELV BMD and appendicular lean mass did not show a good fit (RMSEA = 0.417; CFI = 0.092). The results showed that PELV BMD at T1 positively predicted T2 appendicular lean mass, while PELV BMD at T2 positively predicted T3 appendicular lean mass (Figure 2(b)). Moreover, appendicular lean mass at T1 positively predicted T2 PELV BMD, and appendicular lean mass at T2 positively predicted T3 PELV BMD (Figure 2(b)).

### 4.7. Skull Osteoblasts and Femur Osteoblasts Exert Different Influences on Myoblasts

Myoblasts, such as murine C2C12 myoblasts, are usually utilized for *in vitro* studies of muscle mass in sarcopenia [24]. However, osteoblasts are critical in maintaining BMD [25, 26]. Therefore, the correlation of BMD and muscle mass (sarcopenia) could involve the interaction of osteoblasts and myoblasts.

Our recent study has indicated that skull BMD negatively correlates with ASM mass, whereas BMDs throughout the rest of the body are positively associated with ASM mass in male middle-aged and elderly Chinese individuals [9]. Our current study indicated that WBTOT BMD could temporally and positively predict appendicular lean mass. Femur is the longest and strongest bone of the body [27], suggesting that the BMD of the femur plays a crucial role in WBTOT BMD except skull BMD. Thus, the effects of skull osteoblasts and femur osteoblasts on myoblasts were investigated.

To identify the effects of different osteoblasts on myoblasts, we detected the proliferation, apoptosis, and differentiation of myoblasts. The results showed that a culture medium of primary mice skull osteoblasts enhanced the proliferation of C2C12 cells, while a culture medium of primary mice femur osteoblasts had no effect on the proliferation of C2C12 cells (Figure 3(a)). Treatments of a culture media of primary mice femur osteoblasts and a culture medium of primary mice skull osteoblasts only slightly induced the apoptosis of C2C12 cells (Figure 3(b)), suggesting that the culture medium of primary mice femur osteoblasts and the culture medium of primary mice skull osteoblasts also had no effect on C2C12 cell apoptosis.

Next, the effects of skull osteoblasts and femur osteoblasts on the differentiation of myoblasts were explored. qPCR analysis showed that mRNA levels of myoblast differentiation makers Myog and Myf5 were increased in C2C12 cells cultured with differential medium (DM) compared with those in C2C12 cells cultured with normal culture medium (CM) (Figure 4(a)). Moreover, treatment with a culture medium of primary mice femur osteoblasts increased the mRNA levels of Myog and Myf5 in C2C12 cells, and the addition of culture medium of primary mice femur osteoblasts to DM further enhanced the effect of DM on Myog and Myf5 mRNA expression (Figure 4(a)). In contrast, treatment with a culture medium of primary mice skull osteoblasts reduced the mRNA levels of Myf5 and Myog, and the addition of a culture medium of primary mice skull osteoblasts to DM abolished the effect of DM on Myog and Myf5 mRNA expression (Figure 4(a)).

Similarly, protein levels of the myoblast differentiation makers Myog and myosin heavy chain 6 (MYH6) were increased in C2C12 cells cultured with DM compared with those in C2C12 cells cultured with CM (Figure 4(b)). Treatment with a culture medium of primary mice femur osteoblasts upregulated the protein expression levels of Myog and MYH6, while the addition of a culture medium of primary mice femur osteoblasts to DM further enhanced the effect of DM on Myog and MYH6 protein expression levels (Figure 4(b)). However, treatment with a culture medium of primary mice skull osteoblasts reduced the protein levels of Myog and MYH6, and the addition of a culture medium of primary mice skull osteoblasts to DM abolished the effect of DM on Myog and MYH6 protein expression (Figure 4(b)).

As Myog is associated with oxidative stress, the markers of oxidative stress, including MDA, GSH, and SOD, were detected in C2C12 cells. We showed that the MDA level was decreased, whereas the levels of GSH and SOD were increased, in C2C12 cells cultured with DM compared with those in C2C12 cells cultured with CM (Figures 4(c)–4(e)). Moreover, treatment with a culture medium of primary mice femur osteoblasts reduced the MDA level but elevated the levels of GSH and SOD, while the addition of culture medium of primary mice femur osteoblasts to DM further enhanced the effect of DM on the levels of MDA, GSH, and SOD (Figures 4(c)–4(e)). Nevertheless, treatment with a culture medium of primary mice skull osteoblasts increased the MDA level but decreased the levels of GSH and SOD, and the addition of culture medium of primary mice skull osteoblasts to DM abolished the effect of DM on the levels of MDA, GSH, and SOD (Figures 4(c)–4(e)). These data suggested that primary mice femur osteoblasts, but not primary mice skull osteoblasts, induce the differentiation of C2C12 cells.

### 4.8. Exosomes Derived from Skull Osteoblasts or Femur Osteoblasts Exert Different Effects on Myoblasts

As exosomes mediate the communication among different cells and organs, the effects of exosomes derived from different osteoblasts on myoblasts were examined. Both skull osteoblast–derived exosomes and femur osteoblast–derived exosomes had a cup-shaped morphology with a size of 50–150 nm as detected by TEM and NanoSight analysis (Figures 5(a) and 5(b)). Detection of exosomal markers CD63 and CD81 by WB confirmed that extracellular vesicles isolated from the culture medium of skull osteoblasts or femur osteoblasts were exosomes (Figure 5(c)). Next, C2C12 cells were incubated with exosomes derived from skull osteoblasts or femur osteoblasts, and cell proliferation, apoptosis, and differentiation were recorded. Compared with C2C12 cells culture without exosomes, both skull osteoblast–derived exosomes and femur osteoblast–derived exosomes had no effect on the proliferation and apoptosis of C2C12 cells (Figures 5(d) and 5(e)). Femur osteoblast–derived exosomes increased the protein levels of Myog and MYH6 in C2C12 cells cultured with DM (Figure 5(f)). In contrast, skull osteoblast–derived exosomes decreased the protein levels of Myog and MYH6 in C2C12 cells cultured with DM (Figure 5(f)). These results suggested that femur osteoblast–derived exosomes enhanced the differentiation of myoblasts, whereas skull osteoblast–derived exosomes suppressed this process.

### 4.9. Levels of lncRNA TUG1 and DANCR in Skull and Femur Osteoblast–Secreted Exosomes

So far, the role of exosomal lncRNA TUG1 and DANCR from osteoblasts in myoblasts has been unclear. First, the levels of lncRNA TUG1 and DANCR in osteoblast-secreted exosomes and osteoblasts were detected by qPCR. We found that the level of lncRNA TUG1 in skull osteoblast–secreted exosomes was lower than that in femur osteoblast–secreted exosomes (Figure 6(a)). In contrast, the level of lncRNA DANCR in skull osteoblast–secreted exosomes was higher than that in femur osteoblast–secreted exosomes (Figure 6(b)). Moreover, the level of lncRNA TUG1 in skull osteoblasts was higher than that in femur osteoblasts, while the level of lncRNA DANCR in skull osteoblasts was lower than that in femur osteoblasts (Figures 6(c) and 6(d)), suggesting that the enrichment of lncRNA TUG1 or DANCR in osteoblast-secreted exosomes was negatively related to its expression in osteoblasts. These data indicated that osteoblast-secreted exosomes might exert different influences on myoblasts depending on the levels of exosomal lncRNA TUG1 and DANCR.

### 4.10. Skull and Femur Osteoblast–Secreted Exosomes Alter the Levels of lncRNA TUG1 and DANCR in Myoblasts

To identify whether osteoblast-derived exosomes regulate the levels of lncRNA TUG1 and DANCR in myoblasts, the levels of lncRNA TUG1 and DANCR in C2C12 cells were detected by qPCR after the incubation with osteoblast-derived exosomes. The results revealed that skull osteoblast–secreted exosomes increased the level of lncRNA DANCR in C2C12 cells, while femur osteoblast–secreted exosomes upregulated the level of lncRNA TUG1 in C2C12 cells (Figures 7(a) and 7(b)). These results suggested that lncRNA TUG1 and DANCR in osteoblast-secreted exosomes might contribute to myoblast functions.

### 4.11. lncRNA TUG1 and DANCR Play Different Roles in Myoblasts

To determine the effects of lncRNA TUG1 and DANCR on myoblasts, lncRNA TUG1 and DANCR were overexpressed by transfection of expression vectors into C2C12 cells followed by detections of cell proliferation, apoptosis, and differentiation. Consistent with the results of exosomes incubation, overexpression of lncRNA TUG1 or DANCR had no effect on C2C12 cell proliferation and apoptosis (Figures 8(a) and 8(b)). lncRNA TUG1 overexpression increased and overexpression of lncRNA DANCR reduced the protein levels of Myog and MYH6 in differential C2C12 cells (Figure 8(c)). These results suggested that lncRNA TUG1 enhanced the differentiation of myoblasts, whereas lncRNA DANCR suppressed this process.

### 4.12. lncRNA TUG1 and DANCR Exert Different Effects on *Myog* Expression via Myf5 in Myoblasts

The prediction of RNA–protein binding by RPISEQ showed that both lncRNA TUG1 and DANCR had high binding probability with myogenic transcription factor Myf5 (Supplementary Figure S1). Thus, RIP assay was performed to identify the interaction between Myf5 and lncRNA TUG1 or DANCR. The results of RIP showed the enrichment of lncRNA TUG1 and DANCR by Myf5 protein, suggesting that lncRNA TUG1 and DANCR were associated with Myf5 protein in C2C12 cells (Figure 9(a)).

Furthermore, luciferase reporter gene assay demonstrated that the luciferase activity of C2C12 cells transfected with plasmids containing the *Myog* gene promoter was increased by the transfection of the lncRNA TUG1 expression vector compared with that of cells cotransfected with plasmids containing the *Myog* gene promoter and a blank expression vector, and transfection of the Myf5 expression vector enhanced the effect of the lncRNA TUG1 expression vector (Figure 9(b)). The luciferase activity of C2C12 cells transfected with plasmids containing the *Myog* gene promoter was decreased by the transfection of the lncRNA DANCR expression vector compared with that of cells cotransfected with plasmids containing the *Myog* gene promoter and a blank expression vector, and transfection of the Myf5 expression vector reversed the effect of the lncRNA DANCR expression vector (Figure 9(b)). These data suggested that lncRNA TUG1 promoted the transcription of the *Myog* gene by Myf5, whereas lncRNA DANCR suppressed the transcription of the *Myog* gene via Myf5.

### 4.13. lncRNA TUG1 and DANCR Regulate *Myog* Expression via Modifying Nuclear Translocation of Myf5 in Myoblasts

As Myf5 is a transcription factor, lncRNA TUG1 and DANCR might affect the binding between Myf5 and the *Myog* gene promoter. To prove this hypothesis, ChIP followed by qPCR was performed using Myf5 antibody. The results indicated that Myf5 bound to the *Myog* gene promoter in C2C12 cells (Figures 9(c) and 9(d)). Furthermore, overexpression of lncRNA TUG1 dramatically facilitated the binding of Myf5 to the *Myog* gene promoter in C2C12 cells (Figure 9(c)). In contrast, lncRNA DANCR overexpression suppressed the association of Myf5 with the *Myog* gene promoter in C2C12 cells (Figure 9(c)). These results suggested that lncRNA TUG1 and DANCR exerted opposite effects on the transcription of *Myog* gene through modifying the binding of Myf5 to the *Myog* gene promoter.

In addition, the results of IHC showed that overexpression of lncRNA TUG1 enhanced the nuclear translocation of Myf5, whereas lncRNA DANCR overexpression inhibited the nuclear translocation of Myf5 in C2C12 cells (Figure 9(d)). Thus, lncRNA TUG1 might transport Myf5 into the nucleus, while lncRNA DANCR is mainly located in the cytoplasm after associating with Myf5. These data suggest that lncRNA TUG1 and DANCR regulate the transcription of *Myog* gene through modifying the binding of Myf5 to the *Myog* gene promoter by affecting the nuclear translocation of Myf5 as transporters in C2C12 cells.

## 5. Discussion

In this study, the cross-lagged models indicated that LDL-C positively predicted appendicular lean mass and negatively predicted HEAD BMD. WBTOT BMD, LS BMD, and PELV BMD temporally and positively predicted appendicular lean mass, while appendicular lean mass temporally and positively predicted WBTOT BMD, LS BMD, and PELV BMD. In addition, the present study investigated mechanisms by which different osteoblasts exerted different influences on muscle. First, primary mice femur osteoblasts, but not primary mice skull osteoblasts, induced the differentiation of C2C12 cells through exosomes. Second, the level of lncRNA TUG1 was decreased, and the level of lncRNA DANCR was increased in skull osteoblast–secreted exosomes, whereas the level of lncRNA TUG1 was increased and the level of lncRNA DANCR was decreased in femur osteoblast–secreted exosomes. Moreover, lncRNA TUG1 enhanced the differentiation of myoblasts, whereas lncRNA DANCR suppressed this process through regulating *Myog* expression via modifying the nuclear translocation of Myf5.

Several studies have indicated that albumin, LDL-C, and TSH are related to sarcopenia or muscle mass. For instance, serum albumin level is significantly lower in patients with sarcopenia than in healthy controls [28, 29]. Sarcopenia is associated with urinary albumin level in diabetic patients [30]. Moreover, serum albumin is positively related to lean mass and appendicular lean mass in healthy young individuals [31]. Meanwhile, the LDL-C level is reduced in older people with low muscle mass [32], and serum TSH level has a U-shaped correlation with sarcopenia in older adults [33]. In addition, albumin, LDL-C, and platelet distribution are associated with BMD. A recent study has demonstrated that BMD is negatively related to urine albumin [34]. LDL-C is negatively associated with BMD [35, 36]. Furthermore, TSH suppression leads to a decrease in BMD [37, 38]. Our results indicated that LDL-C positively predicted appendicular lean mass. Thus, bone may exert influences on muscle, combined with LDL-C, in sarcopenia.

The temporal association between sarcopenia or muscle mass with BMD remains unknown. To date, few studies have shown the temporal correlation of sarcopenia or muscle mass and BMD. For example, the increase in appendicular lean mass is temporally associated with increased total hip BMD over 5 years [39]. For the first time, the current study demonstrated that WBTOT BMD, LS BMD, and PELV BMD were able to temporally and positively predict appendicular lean mass. In turn, appendicular lean mass was also able to temporally and positively predict WBTOT BMD, LS BMD, and PELV BMD. Therefore, the present study expanded the knowledge of the temporal association between sarcopenia and muscle mass with BMD.

To date, the knowledge on mechanisms by which bone tissues/osteoblasts exert influence on muscle tissues/myoblasts is still limited. Exosomes mediate the communication among different cells and organs [14]. A previous study has demonstrated that C2C12 myoblasts–derived exosomes facilitate osteogenic differentiation of MC3T3-E1 cells through delivering miR-27a-3p [40]. Nevertheless, the role of exosomes derived from osteoblasts in myoblasts is largely unknown. Several studies have revealed the influences of osteoblast-derived exosomes on other cells or organs. For example, osteoblast-derived exosomes enhance the calcification of vascular smooth muscle cells (VSMCs) [41]. miR-139-5p in senescent osteoblast–secreted exosomes promotes senescence and apoptosis of vascular endothelial cells through targeting T-box transcription factor 1 (TBX1) in endothelial cells [42]. Moreover, exosomes from osteoblasts inhibit T-cell activity [43]. Previous studies have also revealed the effect of osteoblast secretions on myoblasts or muscle cells. For instance, osteoblast-derived OGN may play a role in regulating muscle mass [13]. Furthermore, osteoblasts secrete active osteocalcin to indirectly regulate myoblast functions [44]. However, the role of osteoblast-derived exosomes in myoblasts or muscle cells has not been reported. Therefore, this study revealed the effects of osteoblast-derived exosomes on myoblast differentiation for the first time.

Exosomes could mediate long-distance communication and cooperative regulatory network among different cells and organs as vectors to carry lncRNA in a variety of diseases. For example, bladder cancer cell–derived exosomal lncRNA lymph node metastasis-associated transcript 2 (LNMAT2) enhances lymphatic metastasis through upregulating prospero homeobox 1 (PROX1) expression in lymphatic endothelial cells [45]. In addition, carcinoma-associated fibroblast-secreted exosomal lncRNA H19 improves the stemness and chemoresistance of colorectal cancer (CRC) by targeting miR-141 in CRC cells [46]. However, knowledge on the roles of exosomal lncRNA TUG1 and DANCR is limited. Only one study has indicated that exosomal lncRNA TUG1 derived from cervical cancer cell suppresses apoptosis of vascular endothelial cells [47]. To date, no studies have demonstrated the effect of exosomal lncRNA DANCR. Thus, the results of this study could expand the knowledge on the roles of exosomal lncRNA TUG1 and DANCR.

Previous studies have found that lncRNA TUG1 promotes the osteogenic differentiation, whereas lncRNA DANCR inhibits osteogenic differentiation via the Wnt/*β*-catenin pathway [18, 19]. lncRNA TUG1 upregulates fibroblast growth factor 1 (FGF1) expression to enhance endothelial differentiation via sponging miR-143 in adipose-derived stem cells [48]. In contrast, lncRNA DANCR suppresses odontoblast differentiation through increasing c-Cbl level by sponging miR-216a [15]. Therefore, both lncRNA TUG1 and DANCR play critical roles in cell differentiation. However, the roles of lncRNA TUG1 and DANCR in myoblasts differentiation have not been reported. This study revealed the effects of lncRNA TUG1 and DANCR on the differentiation of myoblasts, which were consistent with previous studies.

Our study indicated that lncRNA TUG1 regulated the transcription of *Myog* gene through modifying the binding of Myf5 to the *Myog* gene promoter by affecting the nuclear translocation of Myf5 as a transporter. Except as a transporter of Myf5 to regulate the binding of Myf5 to the *Myog* gene promoter, lncRNA TUG1 might modify the binding of Myf5 to the *Myog* gene promoter directly. Numerous studies have revealed that lncRNAs could regulate the transcription of target genes through recruiting transcription factors to the promoter of target genes [49, 50]. A previous study demonstrated that lncRNA TUG1 represses Kruppel-like factor 2 (KLF2) expression by interacting with polycomb repressive complex 2 (PRC2) and recruiting it to the *KLF2* gene promoter [51]. Thus, we assume that lncRNA TUG1 might facilitate the binding between Myf5 and the *Myog* gene promoter through recruiting Myf5 to the *Myog* promoter after transporting Myf5 into nucleus.

However, there are several limitations in the current study. First, more patients should be recruited to improve the accuracy of the cross-lagged models utilized for analyzing the temporal association between BMD and muscle mass. Second, data on the grip strength and walking speed of patients should be collected in a future study. Third, in vivo experiments should be performed to certify mechanisms by which exosomal lncRNA TUG1 and DANCR derived from different osteoblasts regulate myoblasts.

## 6. Conclusions

In summary, cross-lagged models indicated that LDL-C positively predicted appendicular lean mass. WBTOT BMD, LS BMD, and PELV BMD temporally and positively predicted appendicular lean mass, while appendicular lean mass in turn temporally and positively predicted WBTOT BMD, LS BMD, and PELV BMD. Moreover, this study revealed that femur osteoblast–derived exosomal lncRNA TUG1 and skull osteoblast–derived exosomal DANCR exerted opposite effects on myoblast differentiation through regulating the transcription of the *Myog* gene by modifying the binding of Myf5 to the *Myog* gene promoter via affecting the nuclear translocation of Myf5 as transporters (Figure 10). Therefore, the results of the present study may provide novel diagnostic biomarkers and therapy targets for sarcopenia.

## Figures and Tables

**Figure 1:** Cross-lagged paths between WBTOT BMD and appendicular lean mass (a) and HEAD BMD and appendicular lean mass (b).

**Figure 2:** Cross-lagged paths between LS BMD and appendicular lean mass (a) and PELV BMD and appendicular lean mass (b).

**Figure 3:** Skull osteoblasts and femur osteoblasts exert different influences on the proliferation and apoptosis of myoblasts. (a) The proliferation rate of C2C12 cells detected by CCK8 array. (b) Representative images of flow cytometric apoptosis assay in C2C12 cells. The bar graph shows the quantification of apoptotic cell number in each group. *N* = 3. ^∗^*P* < 0.05.

**Figure 4:** Skull osteoblasts and femur osteoblasts exert different influences on the differentiation of myoblasts. (a) The levels of Myog and Myf5 mRNA in C2C12 cells detected by qPCR. (b) The protein levels of Myog and MYH6 in C2C12 cells detected using WB. The bar graph shows the relative levels of Myog and MYH6 in each group. (c) The level of MDA in C2C12 cells. (d) The level of GSH in C2C12 cells. (e) The level of SOD in C2C12 cells. CM: C2C12 cell culture medium; DM: differential medium. *N* = 3. ^∗^*P* < 0.05 and ^∗∗^*P* < 0.01.

**Figure 5:** Exosomes derived from skull osteoblasts or femur osteoblasts exert different effects on myoblasts. (a) Representative images of purified skull osteoblast– or femur osteoblast–derived exosomes detected by TEM. Scale bars: 100 nm. (b) Purified exosomes derived from skull osteoblasts or femur osteoblasts were identified by nanoparticle tracking analysis. (c) WB analysis of exosomal markers CD63 and CD81 in exosomes derived from skull osteoblasts or femur osteoblasts. (d) The proliferation rate of C2C12 cells detected by CCK8 array. (e) Representative images of flow cytometric apoptosis assay in C2C12 cells. The bar graph shows the quantification of apoptotic cell number in each group. (f) The protein levels of Myog and MYH6 in C2C12 cells detected using WB. The bar graph shows the relative levels of Myog and MYH6 in each group. CM: C2C12 cell culture medium; DM: differential medium; Exo, exosomes. *N* = 3. ^∗^*P* < 0.05 and ^∗∗^*P* < 0.01.

**Figure 6:** Levels of lncRNA TUG1 and DANCR in skull and femur osteoblast–secreted exosomes. (a) The level of lncRNA TUG1 in exosomes derived from skull osteoblasts or femur osteoblasts. (b) The level of lncRNA DANCR in exosomes derived from skull osteoblasts or femur osteoblasts. (c) The level of lncRNA TUG1 in skull osteoblasts or femur osteoblasts. (d) The level of lncRNA DANCR in skull osteoblasts or femur osteoblasts. Exo: exosomes. *N* = 3. ^∗^*P* < 0.05 and ^∗∗^*P* < 0.01.

**Figure 7:** Skull and femur osteoblast–secreted exosomes alter the levels of lncRNA TUG1 and DANCR in myoblasts. (a) The level of lncRNA TUG1 in C2C12 cells treated with exosomes derived from skull osteoblasts or femur osteoblasts. (b) The level of lncRNA DANCR in C2C12 cells treated with exosomes derived from skull osteoblasts or femur osteoblasts. Exo: exosomes. *N* = 3. ^∗∗^*P* < 0.01.

**Figure 8:** lncRNA TUG1 and DANCR play different roles in myoblasts. (a) The proliferation rate of C2C12 cells detected by CCK8 array. (b) Representative images of flow cytometric apoptosis assay in C2C12 cells. The bar graph shows the quantification of apoptotic cell number in each group. (c) The protein levels of Myog and MYH6 in C2C12 cells detected using WB. The bar graph shows the relative levels of Myog and MYH6 in each group. CM: C2C12 cell culture medium; DM: differential medium; Vec: expression vector; OE: overexpression. *N* = 3. ^∗^*P* < 0.05 and ^∗∗^*P* < 0.01.

**Figure 9:** lncRNA TUG1 and DANCR regulate Myog expression via modifying nuclear translocation of Myf5 in myoblasts. (a) The level of lncRNA TUG1 and DANCR binding to Myf5 protein detected by RIP assay. (b) *Myog* gene promoter activity analyzed by relative luciferase reporter activities in C2C12 cells transfected with lncRNA TUG1 expression vector, lncRNA DANCR expression vector, or Myf5 expression vector. (c) Quantification of Myf5 occupancy on the *Myog* gene promoter by ChIP-qRT-PCR in C2C12 cells transfected with lncRNA TUG1 expression vector or lncRNA DANCR expression vector. (d) Representative images of C2C12 cells staining by Myf5 antibody using IF. The bar graph shows the quantification of mean fluorescence intensity (MFI) of red in the nucleus. Bar = 100 *μ*m. OE: overexpression. *N* = 3. ^∗^*P* < 0.05 and ^∗∗^*P* < 0.01.

**Figure 10:** Schematic diagram of molecular mechanisms. The cross-lagged models indicated that LDL-C positively predicted appendicular lean mass. WBTOT BMD, LS BMD, and PELV BMD temporally and positively predicted appendicular lean mass, while appendicular lean mass in turn temporally and positively predicted WBTOT BMD, LS BMD, and PELV BMD. Moreover, this study revealed that femur osteoblast–derived exosomal lncRNA TUG1 and skull osteoblast–derived exosomal DANCR exerted opposite effects on myoblast differentiation through regulating the transcription of *Myog* gene by modifying the binding of Myf5 to the *Myog* gene promoter via affecting the nuclear translocation of Myf5 as transporters.

**Table 1:** Clinicopathological characteristics of patients with sarcopenia.

Characteristics	Mean value		
	T1	T2	T3
Age (years)	51.57 ± 8.88	52.61 ± 8.88	53.65 ± 8.90
Weight (kg)	72.70 ± 8.39	72.53 ± 8.3	72.67 ± 8.63
Height (cm)	170.50 ± 5.70	170.48 ± 5.69	170.34 ± 5.62
Body mass index (BMI kg/m^2^)	25.00 ± 2.56	24.95 ± 2.54	25.03 ± 2.60

**Table 2:** Descriptive statistics.

Characteristics	Mean value		
	T1	T2	T3
Appendicular lean mass	8.07 ± 0.79	7.96 ± 0.79	7.92 ± 0.78
WBTOT BMD	1.12 ± 0.09	1.12 ± 0.09	1.11 ± 0.091
Head BMD	2.19 ± 0.27	2.17 ± 0.26	2.11 ± 0.32
LS BMD	1.00 ± 0.14	1.00 ± 0.15	1.00 ± 0.15
PELV BMD	1.24 ± 0.17	1.24 ± 0.17	1.22 ± 0.17
Albumin-1 (*μ*g/mL)	43.47 ± 2.23		
FBS (*μ*g/mL)	5.29 ± 1.10		
LDL-C (*μ*g/mL)	2.94 ± 0.74		
TSH (*μ*g/mL)	1.77 ± 1.18		
Platelet distribution width	13.44 ± 2.23		

## Data Availability

Data and material are available upon request.

## Supplementary Materials

Supplementary Materials Supplementary Figure S1: prediction of binding probability between lncRNA TUG1 or DANCR and Myf5. Prediction of binding probability between lncRNA TUG1 (A) or DANCR (B) and Myf5 using RPISEQ (http://pridb.gdcb.iastate.edu/RPISeq/index.html).
